The article "A case series on the effect of lidocaine injection on camptocormia in Parkinson disease: Determination of injection site using muscle hardness tester" was published in 2025. Journal: Medicine (Baltimore).

# A case series on the effect of lidocaine injection on camptocormia in Parkinson disease: Determination of injection site using muscle hardness tester

**DOI:** 10.1097/MD.0000000000043149

**Published:** 2025-07-25

**Authors:** Katsunori Yokoi, Masashi Tsujimoto, Keisuke Suzuki, Akinori Takeda, Kentaro Horibe, Akiko Yamaoka, Eriko Imai, Kazunori Imai, Masahisa Katsuno, Yutaka Arahata

**Affiliations:** a Department of Neurology, National Center for Geriatrics and Gerontology, Obu, Aichi, Japan; b Department of Neurology, Nagoya University Graduate School of Medicine, Nagoya, Japan; c Innovation Center for Translational Research, National Center for Geriatrics and Gerontology, Obu, Aichi, Japan.

**Keywords:** case report, lidocaine injection, muscle hardness tester, Parkinson disease

## Abstract

**Rationale:**

Camptocormia is a debilitating postural abnormality associated with Parkinson disease (PD), significantly impairing the daily lives of affected patients. Treatment options remain inconsistent, with lidocaine injections emerging as a potential therapy. However, the lack of standardized protocols hinders their widespread application. The present study aimed to introduce a novel method using a muscle hardness tester to objectively determine optimal injection sites.

**Patient concerns:**

Patients presented with postural abnormalities characterized by forward flexion, which interfered with daily activities and reduced their quality of life.

**Diagnoses:**

Camptocormia associated with PD was diagnosed based on clinical assessment and radiographic evaluation.

**Interventions:**

Lidocaine injections were administered to 4 patients with PD and camptocormia. Injection sites were determined based on muscle hardness measurements obtained using a muscle hardness meter. A total of 20 mL of 1% lidocaine, distributed as 2.5 mL per injection at 8 sites with the highest muscle hardness values, was administered daily for 5 consecutive days. The postural evaluation was conducted using established criteria, assessing both lower and upper flexion. Radiographic parameters, including lumbar lordosis, thoracic kyphosis, and sagittal vertical axis, were also evaluated. Radiographic assessments were performed on days 1, 5, and 1 month postinjection.

**Outcomes:**

Post-treatment assessments, including spinal flexion measurements and subjective symptom evaluations, demonstrated symptomatic improvement in all cases, particularly in sagittal vertical axis, a key indicator of postural alignment.

**Lessons:**

Our method offers a reproducible approach for enhancing lidocaine injection efficacy. Given its transient effects, repeated administration was necessary. Future studies should focus on refining dosing regimens and expanding case numbers to establish long-term efficacy and optimize treatment strategies. The widespread adoption of this therapy may significantly benefit patients with PD affected by camptocormia.

## 1. Introduction

Parkinson disease (PD) is the second most common neurodegenerative disease after Alzheimer disease. Its frequency increases with age, with a reported prevalence of 3.1% in individuals aged over 75 years and 4.5% in those aged over 85 years.^[1,2]^ Patients with Parkinson and other Parkinson disease-related conditions exhibit postural abnormalities such as camptocormia and cervical dropsy.^[3]^ Postural disorders often affect the basic activities of daily living, such as eating and walking. The prevalence of camptocormia in patients with PD ranges from 3% to 18%, and both central and peripheral mechanisms potentially contribute to its etiology.^[4]^ Notably, camptocormia is often refractory and has been suggested to be associated with dystonia.^[5]^ In addition to neurogenic mechanisms, camptocormia may be induced by medications commonly used in PD treatment, including dopaminergic agents and antipsychotics. These drug-induced cases have been reported to improve following dose reduction or discontinuation.^[6]^

The cause of postural disorders remains unconfirmed, although factors such as negative dystonia and other effects have been suggested. Moreover, no definitive treatment has been established to date.^[7]^ Deep brain stimulation therapy and botulinum toxin in the internal globus pallidus may be effective in improving camptocormia in some patients.^[8,9]^ Additionally, botulinum toxin use carries the potential for prolonged side effects. In light of this, a few institutions in Japan have effectively treated postural disorders by injecting lidocaine into tense muscles in patients with cervical dropsy or camptocormia.^[10,11]^ Currently, treatment methods vary by facility, with no established protocols or universally accepted standard treatment in Japan or abroad.

Previously, injection sites were identified by manual palpation, which is a subjective method with limited reproducibility. Electromyography (EMG)-guided injections offer enhanced precision; however, they are invasive and often painful.^[11]^ To address these limitations, our hospital introduced a muscle hardness meter to objectively determine the injection site and used lidocaine for the injection. The present report introduces our method and its effectiveness, advocating its broader adoption to benefit patients.

## 2. Participants and methods

### 2.1. Indications for lidocaine injection

The inclusion criteria based on indications for lidocaine injections were as follows: a diagnosis of PD; camptocormia significantly impairing daily activities; and in drug-induced cases, the causative drug cannot be discontinued after attempting to adjust the drug. The exclusion criteria included camptocormia due to other diseases, inability to understand treatment due to cognitive decline, and inability to undergo inpatient treatment and rehabilitation for any reason. The treatment paradigm used for the 4 patients with PD in the camptocormia analysis is outlined in Figure 1A.

**Figure 1.** Lidocaine injection paradigm using a muscle hardness tester (A) and evaluation method (B).

### 2.2. Lidocaine injection protocol

The protocol is depicted in Figure 1A. First, muscle hardness values were determined using a muscle hardness tester (NEUTONE TDM-Z2®) and recorded. As no prior reports have used a muscle hardness meter to determine injection sites, we documented the findings on a self-designed record sheet. Second, 2.5 mL of 1% lidocaine was injected at 8 sites with the highest muscle hardness values. In previous reports, lidocaine was injected at a rate of 2.5 to 5 mL per site, with a total of 5 to 10 mL used; however, in this case, the area to be treated was larger, so the total amount was standardized at 20 mL.^[10,11]^ Third, a follow-up with postinjection rehabilitation was conducted. This rehabilitation focused primarily on promoting an upright posture and reducing muscle stiffness through targeted stretching and physical therapy exercises. Finally, following previous reports, injections were administered daily for 5 days as 1 course.^[10,11]^

### 2.3. Evaluation of camptocormia

Camptocormia was evaluated, as presented in Figure 1B. The criteria for the evaluation and diagnosis of kyphotic postures were implemented following those outlined by Fasano et al.^[12]^ Lower flexion was defined as involuntary flexion of the spine that was at least 30° of flexion at the lumbar vertebral point (LF: LI-Sacrum, hip flexion) and that resolved in the supine position. Upper flexion was defined as involuntary flexion of the spine that was at least 45° of flexion at the thoracic vertebral point (TF: C7 to T12-L1) and resolved in the supine position.^[12]^

We also evaluated the following indices: lumbar lordosis (LL), which is the angle between the L1 and S1 upper endplates; thoracic kyphosis angle (TK), which is the angle between T4 and Th12 superior endplates; and sagittal vertical axis (SVA), which is the horizontal distance between the C7 central vertical line and S1 superior posterior edge. Each of these indices was assessed using radiographs taken on the first day of the injection, on the fifth day, and 1 month later, with the entire vertebrae visible in the standing lateral view. We have summarized the results of each indicator in Table 1.

**Table 1:** Radiographic parameters of comptcormia before and after lidocaine injection and 1 mo later.

		LL	TK	TF	LF	SVA
Case 1	Day 1	1	23	58	20	272.37
	Day 5	1	18	60	18	251.94
	1 mo	5	22	59	4	198.57
Case 2	Day 1	12	33	30	32	247.34
	Day 5	15	37	20	25	185.56
	1 mo	11	31	17	25	205.98
Case 3	Day 1	23	16	13	68	176.83
	Day 5	27	13	0	41	140.81
	1 mo	26	13	5	42	144.01
Case 4	Day 1	9	38	40	25	280.96
	Day 5	10	27	33	16	196.76
	1 mo	7	33	37	19	240.76

Day 1 shows the results of the analysis of the X-ray images taken before the first day of lidocaine injections. Day 5 shows the results of the analysis of the X-ray images taken after the end of the fifth day of consecutive lidocaine injections. 1 mo shows the results of the analysis of the X-ray images taken 1 mo after the 5-d course of lidocaine injections.

LF = lumbar fulcrum, LL = lumbar lordosis, SVA = sagittal vertical axis, TF = thoracic fulcrum, TK = thoracic kyphosis.

LF served as an indicator of abnormal posture, where the lumbar spine and femur were bent upward. TF indicated abnormal posture, where the thoracic spine and lumbar spine were bent downward. LL and TK served as indicators of lumbar spine flexion and thoracic spine flexion, respectively. SVA was used as an indicator of postural disorders to evaluate the flexion of the entire spine, including both the thoracic and lumbar spines, in the standing position. The effects of the injection were determined by comparing these indicators before and after the lidocaine injection. For each of the indicators – LF, TFLL, TH, and SVA – an increase in the numerical value indicated a worsening of posture, whereas a decrease in the numerical value indicated an improvement in posture.

## 3. Results

### 3.1. Case 1

The first case involved a 62-year-old woman with upper camptocormia. The patient had a history of lumbar compression and a right femoral neck fracture. She was diagnosed with PD 5 years prior and initially presented with hand tremors. One year before admission, she developed camptocormia, which did not improve after 6 months of medication adjustment. As part of the drug adjustment, the dose of ropinirole administered was reduced and ultimately discontinued. Upon hospitalization, she underwent lidocaine injection therapy, targeting 8 muscle points with the highest hardness values. After 5 days of treatment, the patient exhibited significant improvements in posture, both subjectively and objectively. Compared to day 1, TK and SVA improved on day 5 (Fig. 2A(a,b)). After 1 month, although LL worsened, LF and SVA improved (Fig. 2A(c)). After the treatment, she said, “I was satisfied with the results of the treatment and my vision has improved compared to before.” She continued to receive lidocaine injections every 3 months to maintain her condition.

**Figure 2.** Time series of whole-body lateral radiographs to assess postural changes associated with treatment interventions. (A) Case 1: Radiographs of the spine were taken on the first day (a), 5 d later (b), and 1 mo later (c) after the injection. (B) Case 2: Radiographs of the spine were taken on the first day (a), 5 d later (b), and 1 mo later (c) after the injection. (C) Case 3: Radiographs of the spine were taken on the first day (a), 5 d later (b), and 1 mo later (c) after the injection. (D) Case 4: Radiographs of the spine were taken on the first day (a), 5 d later (b), and 1 mo later (c) after the injection.

### 3.2. Case 2

The second case involved an 83-year-old man with lower camptocormia. The patient had a history of angina pectoris and lumbar spinal stenosis. He was diagnosed with PD 2 years prior, with gait disturbance as the initial symptom. Camptocormia developed 6 months before hospitalization and remained unresponsive to medication adjustments. The patient underwent lidocaine injection therapy for 5 consecutive days. Compared to the first day, improvements in TF, LF, and SVA were observed on the fifth day (Fig. 2B(a,b)). These improvements were maintained even after 1 month (Fig. 2B(c)). No notable changes in LL or TK were observed during or after treatment. He reported notable symptom relief and agreed to receive another course of injections 3 months later. After the treatment, he said, “My posture has improved, I can walk better, and I can eat more easily.” However, owing to family circumstances, he was unable to continue treatment beyond the second session.

### 3.3. Case 3

The third case involved a 79-year-old woman with lower camptocormia. The patient had a pacemaker owing to a history of cardiac disease. She developed PD 8 years ago and initially presented with tremors. Camptocormia appeared 1 year before hospitalization. After an inpatient stay for medication adjustment, she underwent a 5-day course of lidocaine injections (Fig. 2C(a,b)). Compared with the first day, improvements in TF, LF, and SVA were observed on the fifth day of injections, and this trend was maintained even after 1 month (Fig. 2C(c)). LL and TK values remained stable across all time points. The patient reported subjective symptom relief consistent with objective postural improvement. After 5 days of injections, she said, “I feel good, and it’s easier to eat now.” Since then, she has continued to receive injections at 3-month intervals.

### 3.4. Case 4

The fourth case is a 74-year-old man with postural abnormalities characteristic of both upper and lower camptocormia. Although the patient did not strictly meet the angular criteria for upper or lower camptocormia, his forward-flexed posture was sufficiently severe to interfere with basic daily activities such as walking and eating. Given the clinical impact and similarity in presentation, he was included to test whether the same treatment protocol would be beneficial in borderline cases. He had a history of acute gastritis and was diagnosed with PD 3 months before admission. His symptoms began shortly after the diagnosis was made. The patient received a 5-day course of lidocaine injections upon hospitalization, which led to subjective symptom relief (Fig. 2D(a,b)). Compared to the first day, improvements in TK, TF, LF, and SVA were observed on the fifth day, and this trend was maintained even after 1 month (Fig. 2D(c)). LL showed no appreciable change. After 5 days of injections, he said, “It’s easier to move after the injections, so I want you to keep doing them.” Since then, he has continued to receive regular injections every 3 months, reporting sustained improvements in posture and mobility.

## 4. Discussion

There are few effective treatments for camptocormia, and lidocaine may offer a potential solution. A simple dosing regimen using a muscle hardness meter can be implemented by trained healthcare providers, thus negating the necessity of advanced equipment. However, the effect of this regimen is short-lived and requires repeated administrations every 3 months.^[13]^ Moreover, a standardized treatment protocol for lidocaine injections has not yet been established. Although EMG can be used to identify dystonic sites, it is painful.^[11]^ Therefore, some facilities use a simple method to identify and inject rigid muscles by touch. However, this approach involves many subjective factors, and in our facility, we observed variations in the results depending on the practitioner performing the procedure. Therefore, to address this issue, we used a muscle hardness meter to evaluate and identify injection sites objectively. In this report, we present 4 cases of camptocormia associated with PD, demonstrating the effectiveness of lidocaine injections when using a muscle hardness meter. One case had upper camptocormia, and 2 cases had lower camptocormia. Although 1 case did not fit into either category, it still benefited from the treatment. Although Case 4 did not meet the formal diagnostic thresholds, its inclusion reflects a real-world scenario where patients with significant functional impairment may not fulfill strict angular criteria. This suggests that treatment decisions in clinical practice may benefit from more holistic assessments of a patient’s state that also incorporate symptom burden alongside quantitative measures. This is the first case series of lidocaine injections using a muscle hardness tester to determine the injection site. Notably, while reproducibility of muscle hardness measurements was not evaluated in our study, prior studies have shown the device used to be capable of producing consistent results across multiple cases.^[14]^

In this study, we evaluated the following indices: LL, TK, LF, and SVA. TF and LF are expected to serve as indicators of upper and lower postural disorders, respectively. SVA is expected to be an indicator of overall postural disorders. Although formal minimal clinically important differences for these postural indices have not been established, we considered any consistent improvement, particularly in the SVA, which corresponded with patient-reported relief, to be clinically meaningful. Future studies should aim to define MCID thresholds for spinal alignment parameters in camptocormia to support the quantitative assessment of therapeutic outcomes. Moreover, LL and TK are expected to serve as indicators of vertebral flexion. Evaluation of these indices revealed minimal and inconsistent changes in LL and TK. Specifically, TK showed modest improvement in Cases 1 and 4, whereas LL either worsened or remained unchanged in all cases. These findings suggest that the intervention had minimal effect on spinal curvature, in contrast to more consistent improvements observed in TF, LF, and SVA. However, TF or LF improved in each case, while SVA improved in all cases. Given that no improvements were observed in LL and TK, while TF, LF, and SVA exhibited improvements, this suggests that treatment does not improve vertebral flexion but rather enhances posture and overall balance. Overall, these 4 cases suggest that determining the injection site for lidocaine injections in camptocormia using a muscle hardness meter is an effective approach.

In addition, although we evaluated several indices in this study, only SVA improvement was consistently observed, even in cases with limited TF and LF improvements, such as Case 1. Although we used items employed in orthopedic spine evaluations and conventional neurologic assessments of camptocormia,^[15]^ we observed no significant improvement in any of the items related to spinal flexion. However, SVA exhibited improvements in all cases, suggesting it is the most relevant indicator of subjective improvement in posture and a suitable treatment marker for lidocaine injections.

Camptocormia has been suggested to be associated with dystonia, and botulinum toxin injections are generally considered for treating dystonia.^[16]^ However, botulinum toxin has not been demonstrated to be effective against camptocormia in PD,^[17]^ although it has been suggested to improve the posture in some patients.^[8]^ As observed in this case series, lidocaine is an effective treatment approach, and its effects can last for several months. Therefore, lidocaine serves as a safe and effective approach for treating patients with PD complicated by camptocormia, as it is associated with minimal side effects. However, the reason why the effect of lidocaine lasts for several months, although the active time of the drug is only 30 minutes to 3 hours, has not been identified. The continued recovery, as seen in the ability of a patient to correct their posture, may be attributable to a combination of the continuation of physical rehabilitation and lidocaine injections. Overall, the repetition of this process may induce a learning effect, which contributes to the alleviation of postural abnormalities and improvements in balance and gait.^[15]^

In conclusion, the results of this report suggest that lidocaine injection guided by a muscle hardness meter may be a potential solution for camptocormia; however, this study has limitations. It was a case series study limited to a small sample size and lacked a prospective, single-center, or controlled study using a comparator substance. Therefore, disseminating therapies, accumulating cases, and reporting them in the future is important.

## Author contributions

**Conceptualization:** Yutaka Arahata.

**Data curation:** Katsunori Yokoi, Masashi Tsujimoto, Keisuke Suzuki, Akinori Takeda, Kentaro Horibe, Akiko Yamaoka, Eriko Imai, Kazunori Imai.

**Methodology:** Katsunori Yokoi, Masashi Tsujimoto, Keisuke Suzuki, Masahisa Katsuno.

**Supervision:** Yutaka Arahata.

**Validation:** Yutaka Arahata.

**Writing – original draft:** Katsunori Yokoi.

**Writing – review & editing:** Katsunori Yokoi, Akinori Takeda, Masahisa Katsuno, Yutaka Arahata.
